RETRACTED

# *α*-Cyperone Protects Cardiomyocytes against Oxygen-Glucose Deprivation-Induced Inflammation and Oxidative Stress by Akt/FOXO3a/NF-*κ*B Pathway

**DOI:** 10.1155/2022/8205707

**Published:** 2022-08-29

**Authors:** Feiqun Yao, Qian Zhu

**Affiliations:** ^1^Department of Cardiology, Zhuji People's Hospital of Zhejiang Province, Zhuji, 311800 Zhejiang, China; ^2^Department of Pharmacy, Haining People's Hospital, Haining, 314400 Zhejiang, China

## Abstract

**Objective:**

This study is aimed at investigating the mechanism of *α*-cyperone in oxygen and glucose deprivation- (OGD-) induced myocardial injury.

**Methods:**

Cardiomyocytes were exposed to OGD and then treated with *α*-cyperone. The cell counting kit-8 (CCK-8) assay and flow cytometry were performed to determine cell proliferation and apoptosis, respectively. The expression of inflammatory factors was monitored by quantitative reverse transcription-polymerase chain reaction (qRT-PCR). The profiles of apoptosis-related proteins, inflammatory proteins, and the Akt/FOXO3a/NF-*κ*B pathway were determined by western blot. The phosphorylation of Akt, FOXO3a, and NF-*κ*B was determined by immunofluorescence assay. The superoxide dismutase (SOD) activity and the malondialdehyde (MDA) content were gauged by the colorimetric method, and the reactive oxygen species (ROS) content was measured.

**Results:**

*α*-Cyperone hindered OGD-induced inflammation, oxidative stress, and apoptosis in cardiomyocytes. OGD activated the FOXO3a/NF-*κ*B pathway and hampered the Akt phosphorylation. *α*-cyperone reversed OGD-mediated FOXO3a/NF-*κ*B pathway activation. Treatment with MK-2206 abated the protective effect of *α*-cyperone against OGD-induced myocardial injury. The addition of *α*-cyperone to cardiomyocytes following Bay11-7082 treatment had no conspicuous effect on the viability and apoptosis.

**Conclusions:**

*α*-Cyperone protected cardiomyocytes against OGD-induced inflammation and oxidative stress via the Akt/FOXO3a/NF-*κ*B axis.

## 1. Introduction

Acute myocardial infarction (AMI) is a myocardial ischemic necrosis caused by a dramatic reduction or interruption of coronary blood supply [1]. Myocardial injury after AMI is a very complex pathophysiological process involving inflammatory response, immune response, apoptosis, autophagy, and mitochondrial dysfunction [2]. Over the past few years, the incidence of AMI in China has been rising, accompanied by an increase in mortality [3]. AMI remains a major health threat to humans [4]. Therefore, it is very important to explore new therapeutic strategies and underlying mechanisms for AMI.

*α*-Cyperone is one of the main components of Cyperus rotundus oil and has diversified beneficial biological activities [5]. Related studies have exhibited that *α*-cyperone exerts antidepressant effects by enhancing neuroplasticity in mice through inhibition of SIRT3/reactive oxygen species- (ROS-) mediated NLRP3 inflammasomes [6]. In lipopolysaccharide- (LPS-) treated macrophages, *α*-cyperone exerts its anti-inflammatory effects by inactivating NF-*κ*B to downregulate COX-2 and IL-6 [7]. *α*-Cyperone bridles apoptosis, oxidative stress, and mitochondrial dysfunction in H_2_O_2_-treated SH-SY5Y cells through activation of Nrf2 [8]. Nevertheless, *α*-cyperone's mechanism of action in oxygen and glucose deprivation- (OGD-) induced myocardial injury remains unclear.

RETRACTED

Akt is a serine/threonine kinase that exerts an essential function in cell survival, cell growth, cell proliferation, angiogenesis, vasodilation, and cell metabolism [9]. According to reports, YXC attenuates DOX-induced apoptosis, oxidative stress, and inflammation in cardiomyocytes by motivating the Akt/GSK3*β*/*β*-catenin signaling, whereas Akt inhibitors impede this effect of YXC [10]. Forkhead box O 3a (FOXO3a) is a critical transcription factor that is closely associated with various biological processes such as apoptosis, oxidative stress, autophagy, and inflammation [11]. The Akt signaling pathway phosphorylates FOXO3a to regulate its transcriptional function [12]. For example, FGF-2 abates H_2_O_2_-induced cardiomyocyte apoptosis and protects cardiomyocytes from oxidative stress damage by uplifting phosphorylation of Akt and FOXO3a [13]. Nuclear transcription factor-*κ*B (NF-*κ*B) is a key nuclear transcription factor that is implicated in various pathophysiological processes such as inflammatory response, immune response, oxidative stress, and apoptosis [14]. In hypoxia/reoxygenation (H/R) injury, Ginsenoside Rb3 reduces apoptosis and inflammation in cardiomyocytes by blocking the JNK-mediated NF-*κ*B pathway [15]. There is a regulatory relationship between FOXO3a and NF-*κ*B [16]. In sepsis-induced myocardial injury, miR-29b-3p chokes MAPK activation and NF-*κ*B nuclear translocation by decreasing phosphorylation of FOXO3a, thereby reducing cardiomyocyte apoptosis and inflammation [17]. Nonetheless, the mechanism of action of the Akt/FOXO3a/NF-*κ*B pathway in OGD-induced myocardial injury remains elusive.

The purpose of this study was to investigate the mechanism of *α*-cyclotrione in OGD-induced myocardial injury. We found that *α*-cyperone inhibited OGD-induced cardiomyocyte apoptosis, oxidative stress, and inflammation. *α*-Cyperone inhibits OGD-mediated activation of the FOXO3a/NF-*κ*B pathway by stimulating Akt to reduce the phosphorylation of FOXO3a and NF-*κ*B. In addition, Akt inhibition inhibited the cardioprotective effect of *α*-meliolone against OGD injury, and NF-*κ*B inhibition counteracted the protective effect of *α*-lemonillone against OGD-induced myocardial injury. These findings provide a basis for the prevention and treatment of AMI.

RETRACTED

## 2. Materials and Methods

### 2.1. Cell Culture

The H16 was purchased from Procell (SCC109, Procell, China) and HCM cardiomyocytes were isolated and stored in our lab. Cardiomyocytes were grown in DMEM (Sigma-Aldrich; Merck KGaA) containing 10% FBS (Gibco; Thermo Fisher Scientific, Inc.) and a mixture of 100 U/mL penicillin and streptomycin. The culture medium was maintained in an incubator at 37°C with 5% CO_2_.

### 2.2. The OGD Model Construction

The medium was substituted with a sugar-free DMEM (Gibco; Thermo Fisher Scientific, Inc.) and placed in an anaerobic incubator (95% N_2_ and 5% CO_2_) and maintained at 37°C for six hours to establish an OGD injury model [18]. The *α*-cyperone (>98% purity; Yuan ye Biotech, Shanghai, China) was dissolved in DMSO and diluted to a final concentration of 0.05% DMSO. OGD-induced cardiomyocytes (H16 and HCM) were exposed to *α*-cyperone (15, 30, and 60 *μ*M) for 24 hours. The experiment was divided into the CON, *α*-cyperone (60 *μ*M), OGD, OGD+*α*-cyperone (15 *μ*M), OGD+*α*-cyperone (30 *μ*M), and OGD+*α*-cyperone groups.

### 2.3. The Cell Counting Kit-8 (CCK-8) Assay

The cells were seeded in 96-well culture plates (2 × 10^3^ cells/well), and their viability was assayed using the CCK-8 kit. 10 *μ*L of CCK-8 (Dojindo Molecular Technologies, Kumamoto, Japan) solution was added to each well and incubated at 37°C for one hour. The absorbance at 450 nm was reviewed using a spectrophotometer (Bio-Rad, CA, USA). The formula was calculated as the absorbance value of the experimental group/absorbance value of the control group × 100%.

### 2.4. Flow Cytometry

Cardiomyocyte apoptosis was checked with the Annexin V-FITC/PI kit (Becton, Dickinson and Company) as per the manufacturer's instructions. After experimental processing, cells were collected, rinsed twice by centrifugation in PBS, and dyed with a solution of membrane-linked protein V-FITC (5 *μ*L) and propidium iodide (10 *μ*L) for 15 minutes in the dark at 37°C. Apoptotic levels of cardiomyocytes in each treatment group were determined using flow cytometry (FACScan; BD Biosciences).

### 2.5. Western Blot (WB)

The cells were treated with the RIPA buffer (Beyotime, Shanghai, China), and the cell lysates were centrifuged at 12000 rpm at 4°C for 10 minutes. The protein concentrations were determined by the BCA kit (Beyotime Inst. Biotech, Beijing, China). Equal amounts of protein (30 *μ*g) were separated on 10% SDS-PAGE and then transferred to PVDF membranes. The membranes were blocked with 5% skim milk for two hours at room temperature (RT) and incubated with the anti-Akt (Abcam, 1 : 1000, ab8805, Shanghai, China), anti-pAkt (Abcam, 1 : 1000, ab38449), anti-FOXO3a (Abcam, 1 : 1000, ab109629), anti pFOXO3a (Abcam, 1 : 1000, ab154786), anti-NF-*κ*B (Abcam, 1 : 1000, ab32360), anti-pNF-*κ*B (Abcam, 1 : 1000, ab76302), anti-Bcl2 (Abcam, 1 : 1000, ab32124), anti-Bax (Abcam, 1: 1000, ab32503), anti-C-Caspase3 (Abcam, 1 : 1000, ab32042), anti-iNOS (Abcam, 1 : 1000, ab178945), anti-COX2 (Abcam, 1 : 1000, ab62331), and anti-GAPDH (Abcam, 1 : 1000, ab ab9485) antibodies overnight at 4°C. Subsequently, the membranes were washed with TBST four times and incubated at RT with the horseradish peroxidase- (HRP-) labeled anti-rabbit secondary antibody (1 : 3000) for one hour. The protein bands were then visualized using enhanced chemiluminescence (ECL; Pierce; Thermo Fisher Scientific, Inc.). The quantification of bands was performed by using ImageJ software.

RETRACTED

### 2.6. Quantitative Reverse Transcription-Polymerase Chain Reaction (qRT-PCR)

The total RNA was extracted by the TRIzol reagent (Invitrogen, Carlsbad, CA, USA). RNA concentration was measured by a spectrophotometer. About 4 *μ*g of RNA underwent reverse transcription into cDNA by employing the PrimeScript™ RT Reagent kit (Invitrogen, Shanghai, China) as per the manufacturer's instructions. The primer sequences are as follows: TNF-*α*: forward: 5′-CATCTTCTCAAAATTCGAGTGACAA-3′, reverse: 5′-TGGGAGTAGACAAGGTACAACCC-3′; IL-6: forward: 5′-ACTCACCTCTTTCAGAACGAATTG-3′, reverse: 5′-CCATCTTTGGAAGGTTCAGGTTG-3′; IL-1*β*: forward: 5′-CCGTGGACCTTCCAGGATGA-3′, reverse: 5′-GGGAAGGTCACACACCAGCA-3′; ICAM-1: forward: 5′-GACCAGAGGTTGAACCCCAC-3′, reverse: GCGCCGGAAAGCTGTAGAT-3′ (reverse); VCAM-1: forward: 5′-AGTGGTGGCCTCCTGAATGG-3′, reverse: 5′-CTGTGTCTCCTG TCTCCGCT-3′; MCP1: forward: CAGCCAGATGCAATCAATGCC-3′, reverse: TGGAATCCTGAACCCACTTCT-3′; and GAPDH (endogenous control): forward: 5′-GGAGCGAGATCCCTCCCTCC 3′, reverse: 5′-GGCT GTTGTCATACTTCTCATGG-3′. The qRT-PCR was then performed on the ABI 7500 real-time PCR system (ABI, USA) using the SYBR Green QuantiTect RT-PCR kit (Takara Biotechnology Co., Ltd., Dalian. China) in the 20 *μ*L volume with 40 cycles of denaturation at 95°C for 10 seconds, followed by annealing at 60°C for 30 seconds and extension at 72°C for 30 seconds. Statistics were analyzed using the 2^-*ΔΔ*CT^ method, and each experiment was repeated three times.

### 2.7. Colorimetry

The cells were inoculated in 6-well plates, and the cell supernatant was collected and centrifuged at 1000 rpm for 10 minutes at 4°C to obtain the postcentrifugation supernatant. The superoxide dismutase (SOD) activity and malondialdehyde (MDA) content were gauged using SOD and MDA kits (Nanjing JianCheng Bioengineering Institute).

RETRACTED

### 2.8. Cellular Immunofluorescence

To determine the phosphorylation of Akt, FOXO3a, and NF-*κ*B in cardiomyocytes, cardiomyocytes were flushed three times with PBS and then secured in 4% paraformaldehyde solution for 15 minutes. Next, they were maintained with 0.5% Triton X-100 containing goat serum fluorescently labeled goat anti-rabbit IgG antibody. The slides were observed in the dark phase using an inverted fluorescence microscope.

### 2.9. Determination of ROS

H16 and HCM were seeded in 12-well plates (1 × 10^5^ cells/mL), and intracellular ROS levels were evaluated using the ROS Assay Kit (Beyotime Institute of Biotechnology). The cells were flushed with PBS twice and incubated with 10 *μ*M DCFH-DA (Sigma, St. Louis, MO) at 37°C for 20 minutes. Quantitative analysis was made with the FlowJo TM software (Becton, Dickinson & Company, USA).

### 2.10. Statistics and Analysis

All data were expressed as mean ± standard deviation (SD) and statistically analyzed using SPSS 19.0 (SPSS Inc., Chicago, IL, USA). Differences between the two groups were analyzed using *t* test. The two-sided *P* value less than 0.05 indicated statistically significant difference.

## 3. Results

### 3.1. *α*-Cyperone Mitigated OGD-Induced Cardiomyocyte Apoptosis

To make certain the protective effect of *α*-cyperone on cardiomyocytes, we set up OGD models in H16 and HCM cardiomyocytes and treated OGD-induced cardiomyocytes with different concentrations (15, 30, and 60 *μ*M) of *α*-cyperone for 24 hours. CCK-8 and flow cytometry were adopted to test cardiomyocyte viability and apoptosis. As a result, compared to the CON group, OGD-treated cardiomyocytes exhibited increased apoptosis and reduced viability. *α*-Cyperone declined OGD-mediated cardiomyocytes' apoptosis and restored their proliferative activity concentration dependently. In contrast, the use of 60 *μ*M *α*-cyperone alone did not influence cardiomyocyte viability or apoptosis (Figures 1(a) and 1(b)). As displayed by WB data, OGD treatment boosted the levels of Bax and caspase-3 and tarnished the Bcl-2 profile in cardiomyocytes compared to the CON group. *α*-Cyperone concentration dependently hampered the expression of proapoptotic proteins and elevated the expression of antiapoptotic proteins in OGD-induced cardiomyocytes. Meanwhile, the use of 60 *μ*M *α*-cyperone alone did not affect the expression of Bax and caspase-3 in cardiomyocytes but boosted the expression level of Bcl-2 (Figure 1). These data substantiated that *α*-cyperone suppressed apoptosis and enhanced the viability of cardiomyocytes, alleviating the myocardial injury induced by OGD.

RETRACTED

### 3.2. *α*-Cyperone Eased OGD-Induced Cardiomyocyte Inflammation and Oxidative Stress

qRT-PCR and WB outcomes uncovered that OGD-treated cardiomyocytes harbored increased inflammatory factors (TNF-*α*, IL-6, IL-1*β*, MCP1, ICAM1, and VCAM1) and inflammatory response proteins (COX2, iNOS) compared to the CON group. In parallel, these inflammatory factors and inflammatory proteins were downregulated by *α*-cyperone concentration dependently. In contrast, 60 *μ*M *α*-cyperone alone did not affect the expression of inflammatory factors and inflammatory response proteins in cardiomyocytes (Figures 2(a) and 2(b)). The results of colorimetry and ROS assay disclosed that OGD treatment resulted in elevated ROS levels, amplified MDA contents, and reduced SOD activities in cardiomyocytes compared to the CON group, while *α*-cyperone reversed the effects of OGD concentration dependently. In addition, the application of 60 *μ*M *α*-cyperone alone did not influence the levels of ROS, MDA, or SOD (Figures 2(c)–2(e)). These data concluded that *α*-cyperone eased OGD-induced cardiomyocyte inflammation and oxidative stress.

### 3.3. *α*-Cyperone Inactivated the Akt/FOXO3a/NF-*κ*B Axis in OGD-Treated Cardiomyocytes

To elucidate the underlying mechanisms of *α*-cyperone, the effect of *α*-cyperone on the Akt/FOXO3a/NF-*κ*B pathway was assessed in OGD-mediated cardiomyocytes (H16 and HCM). WB and cellular immunofluorescence revealed that OGD treatment restrained the phosphorylation of Akt and enhanced the phosphorylation of FOXO3a and NF-*κ*B in cardiomyocytes compared to the CON group. However, *α*-cyperone (60 *μ*M) upregulated phosphorylation of Akt and decreased phosphorylation of FOXO3a and NF-*κ*B in OGD-mediated cardiomyocytes. In contrast, the phosphorylation of Akt, FOXO3a, and NF-*κ*B in cardiomyocytes was not affected by 60 *μ*M *α*-cyperone alone (Figures 3(a) and 3(b)). These outcomes confirmed that *α*-cyperone inactivated the Akt/FOXO3a/NF-*κ*B pathway in OGD-treated cardiomyocytes and that the Akt/FOXO3a/NF-*κ*B pathway might exert a dominant role in the attenuation of OGD-mediated myocardial injury by *α*-cyperone.

### 3.4. Attenuating Akt Weakened the Protective Effect of *α*-Cyperone on OGD-Induced Myocardial Injury

To probe the function of Akt in the attenuation of OGD-mediated myocardial injury by *α*-cyperone, OGD-induced HCM cells were exposed to *α*-cyperone (60 *μ*M) for 24 hours followed by the addition of the Akt inhibitor MK-2206. CCK-8 and flow cytometry assays demonstrated that the addition of MK-2206 reduced the viability and intensified apoptosis in the OGD-treated cardiomyocytes. Meanwhile, cardiomyocytes in the OGD+*α*-cyperone (60 *μ*M)+MK-2206 group displayed amplified apoptosis and restrained cell viability compared to the OGD+*α*-cyperone (60 *μ*M) group (Figures 4(a) and 4(b)). WB data testified that the addition of MK-2206 to the OGD group resulted in facilitated expression of Bax and caspase-3 and hampered expression of Bcl-2 in cardiomyocytes. *α*-Cyperone suppressed the increase in proapoptotic proteins and the decrease in antiapoptotic proteins in OGD-treated cardiomyocytes, and the addition of MK-2206 reversed this effect of *α*-cyperone (Figure 4(c)). qRT-PCR and WB results exhibited strengthened expression of inflammatory factors and inflammatory response proteins in cardiomyocytes in the OGD+MK-2206 group by contrast with the OGD group. The addition of MK-2206 attenuated the anti-inflammatory effects of *α*-cyperone in OGD-mediated myocardial injury (Figures 4(d) and 4(e)). The results of colorimetry and ROS detection testified that the addition of MK-2206 in the OGD group caused an increase in ROS levels and MDA contents and a decrease in SOD activity in cardiomyocytes. The addition of MK-2206 attenuated the antioxidative stress effect of *α*-cyperone in OGD-mediated myocardial injury (Figures 4(f) and 4(g)). These data uncovered that Akt inhibition suppressed the protective effect of *α*-cyperone on OGD-induced myocardial injury.

RETRACTED

### 3.5. Attenuating Akt Activated the FOXO3a/NF-*κ*B Pathway

WB and cellular immunofluorescence manifested that MK-2206 dampened Akt phosphorylation, enhanced FOXO3a and NF-*κ*B phosphorylation, and activated the FOXO3a/NF-*κ*B pathway in OGD-treated cardiomyocytes compared to the OGD group. Moreover, the addition of MK-2206 to the OGD+*α*-cyperone (60 *μ*M) group resulted in decreased phosphorylation of Akt and enhanced phosphorylation of FOXO3a and NF-*κ*B in cardiomyocytes (Figures 5(a) and 5(b)). These results signified that inhibition of Akt activated the FOXO3a/NF-*κ*B pathway in OGD-induced injury.

### 3.6. Attenuating NF-*κ*B Counteracted the Protective Effect of *α*-Cyperone on OGD-Mediated Myocardial Injury

To figure out the role of NF-*κ*B in the attenuation of OGD-mediated myocardial injury by *α*-cyperone, OGD-induced HCM cells were treated with *α*-cyperone (60 *μ*M) for 24 hours, followed by the addition of the NF-*κ*B inhibitor Bay11-7082. As indicated by CCK-8 and flow cytometry data, Bay11-7082 increased OGD-treated cardiomyocytes' viability and reduced their apoptosis. Nevertheless, there was no distinct difference in the viability and apoptotic rate of cardiomyocytes between the OGD+Bay11-7082 and OGD+*α*-cyperone (60 *μ*M)+Bay11-7082 groups (Figures 6(a) and 6(b)). WB outcomes uncovered that Bay11-7082 downregulated Bax and caspase-3 and upregulated Bcl-2 in OGD-mediated cardiomyocytes compared to the OGD group. However, there was no significant difference in the expression of Bax, caspase-3, and Bcl-2 in the cardiomyocytes of the OGD+Bay11-7082 and OGD+*α*-cyperone (60 *μ*M)+Bay11-7082 groups (Figure 6(c)). qRT-PCR and WB data revealed that Bay11-7082 declined the expression of inflammatory factors and inflammatory response proteins in cardiomyocytes compared to the OGD group. Meanwhile, there was no substantial difference in the expression of inflammatory factors and inflammatory response proteins in cardiomyocytes in the OGD+Bay11-7082 and OGD+*α*-cyperone (60 *μ*M)+Bay11-7082 groups (Figures 6(d) and 6(e)). The results of colorimetry and ROS detection showed that the OGD+Bay11-7082 group had reduced ROS levels and MDA contents and increased SOD activity in cardiomyocytes in comparison to the OGD group. The contents of ROS, MDA and SOD in cardiomyocytes were almost unchanged after the addition of *α*-cyperone (60 *μ*M) in the OGD+Bay11-7082 group (Figures 6(f) and 6(g)). WB exhibited that Bay11-7082 attenuated NF-*κ*B phosphorylation in OGD-treated cardiomyocytes, but it did not affect the phosphorylation of Akt and FOXO3a. Besides, there was little change in the phosphorylation of Akt, FOXO3a, and NF-*κ*B in cardiomyocytes after the addition of *α*-cyperone (60 *μ*M) in the OGD+Bay11-7082 group (Figure 6(h)). These results validated that inhibition of NF-*κ*B reduced OGD-induced cardiomyocyte inflammation, oxidative stress, and apoptosis and enhanced cardiomyocyte viability. In addition, inhibition of NF-*κ*B counteracted the protective effect of *α*-cyperone against OGD-mediated myocardial injury.

RETRACTED

## 4. Discussion

Pathophysiological changes in AMI include lipid deposition, thrombosis, inflammatory response, cardiomyocyte apoptosis, and mitochondrial dysfunction [19]. AMI can lead to serious myocardial damage and even death, and its high incidence and mortality rates pose a serious threat to people's lives [20]. The present research discovered that *α*-cyperone choked OGD-induced apoptosis, oxidative stress, and inflammatory responses in cardiomyocytes. *α*-Cyperone decreased the phosphorylation of FOXO3a and NF-*κ*B through activation of Akt and restrained OGD-mediated activation of the FOXO3a/NF-*κ*B pathway. We demonstrated for the first time that *α*-cyperone attenuated OGD-induced myocardial injury by inactivating the Akt/FOXO3a/NF-*κ*B pathway.

*α*-Cyperone is the main active ingredient of Cyperus rotundus that has anti-inflammatory effects [21]. Related studies have indicated that *α*-cyperone reduces inflammatory cytokine expression by upregulating SIRT1 to inhibit the NLRP3 and NF-*κ*B pathways, thereby alleviating LPS-induced acute lung injury in mice [22]. *α*-Cyperone hinders nuclear translocation of NF-*κ*B by decreasing phosphorylation of MAPKs, thereby reducing chondrocyte inflammation and extracellular matrix degradation in osteoarthritis (OA) mice [23]. *α*-Cyperone exerts neuroprotective effects by spurring the Akt/Nrf2/HO-1 axis and inactivating NF-*κ*B to decline the production of inflammatory factors TNF-*α*, IL-6, and IL-1*β* in LPS-treated microglia [24]. Here, we discovered that *α*-cyperone exerted a cardioprotective effect in OGD injury, enhancing cardiomyocyte viability and hampered apoptosis concentration dependently.

Akt, also known as protein kinase B (PKB), plays a vital role in cell survival and apoptosis [25]. For example, GRX2 exerts cardioprotective effects by activating the Nrf2 pathway via upregulation of Akt and GSK-3*β* phosphorylation to abate cardiomyocyte apoptosis, oxidative stress, and inflammation in H/R injury [26]. Akt can regulate the activity of FOXO3a, one of the main downstream effectors of Akt [27]. H_2_S dampens DOX-induced apoptosis and oxidative stress in cardiomyocytes by heightening phosphorylation of Akt and FOXO3a, thereby attenuating cardiotoxic effects [28]. Kcnh2 restrains apoptosis and inflammatory responses in cardiomyocytes by enhancing the activity of Akt to reduce the phosphorylation of FOXO3a, thereby easing sepsis-induced cardiac injury [29]. Dysregulated activity of NF-*κ*B, an important intracellular transcription factor, leads to inflammation-related diseases [14]. Plantamajoside ameliorates H/R injury by motivating the Akt/Nrf2/HO-1 pathway and inactivating NF-*κ*B to attenuate apoptosis, oxidative stress, and inflammatory responses in cardiomyocytes [30]. Apigenin curbs oxidative stress and inflammation by activating FOXO3a, a possible suppressor of the NF-*κ*B pathway, to attenuate NF-*κ*B activation, thereby reducing MSNs-induced renal injury [31]. FOXO3a may also be a positive regulator of the NF-*κ*B pathway. In sepsis-induced myocardial injury, GSK-3*β* inhibition blocks NF-*κ*B activation by downregulating *β*-catenin-mediated FOXO3a expression, thereby reducing apoptosis and inflammatory responses in rat cardiomyocytes [32]. Here, we observed that *α*-cyperone decreased the phosphorylation of FOXO3a and NF-*κ*B through activation of Akt and inhibited OGD-mediated FOXO3a/NF-*κ*B pathway activation. The Akt inhibitor MK-2206 activated the FOXO3a/NF-*κ*B pathway by abating the phosphorylation of Akt and upregulating the phosphorylation of FOXO3a and NF-*κ*B. Besides, MK-2206 hindered the myocardial protective effect of *α*-cyperone in OGD injury, while Bay11-7082 counteracted the protective effect of *α*-cyperone against OGD injury.

RETRACTED

The occurrence and development of AMI are closely related to increased oxidative stress and inflammatory response [33]. In AMI, ischemic myocardium produces ROS, and excess ROS damages cell membranes, leading to apoptosis and necrosis [34]. SOD is an important superoxide anion scavenger that provides cytoprotection against free radical damage [35]. MDA is a lipid peroxidation product produced in the metabolism of oxygen radicals in the body, reflecting the damage caused by ROS [36]. The inflammatory response following AMI is frequent, and serum levels of inflammatory cytokines and inflammatory response proteins are notably elevated [37]. The present study uncovered that *α*-cyperone attenuated OGD-induced oxidative stress in cardiomyocytes through upregulation of SOD and downregulation of ROS and MDA. *α*-Cyperone curbed the OGD-induced inflammatory response in cardiomyocytes by declining the expression of inflammatory cytokines and inflammatory response proteins. Together, these data substantiate that *α*-cyperone protects cardiomyocytes from OGD damage by mitigating inflammatory response and oxidative stress.

Overall, our study demonstrates that *α*-cyperone exerts a cardioprotective effect by hindering the Akt/FOXO3a/NF-*κ*B pathway to suppress OGD-induced apoptosis, oxidative stress, and inflammation in cardiomyocytes. Inhibition of Akt motivates the FOXO3a/NF-*κ*B pathway and weakens the cardioprotective effect of *α*-cyperone in OGD injury. Besides, inhibition of NF-*κ*B eases the inflammatory response in OGD-induced cardiomyocytes and counteracts *α*-cyperone-mediated myocardial protection. The findings of this research provide new ideas and targets for the prevention and treatment of AMI.

## Figures and Tables

**Figure 1:** *α*-Cyperone alleviated OGD-induced cardiomyocyte apoptosis. Cardiomyocytes were treated with different concentrations (15, 30, and 60 *μ*M) of *α*-cyperone for 24 hours after OGD induction. (a) Detection of cardiomyocyte viability was made using the CCK-8 assay. (b) Percentage of apoptosis in cardiomyocytes was determined with flow cytometry. The profiles of apoptosis-related proteins were checked by WB. All experiments were repeated three times and data were expressed as mean ± SD; ^∗^*P* < 0.05 (vs. CON), ^∗∗^*P* < 0.01, ^∗∗∗^*P* < 0.001, and ^∗∗∗∗^*P* < 0.0001. ^&^*P* < 0.05 (vs. OGD), ^&&^*P* < 0.01, ^&&&^*P* < 0.001, and ^&&&&^*P* < 0.0001.

RETRACTED

**Figure 2:** *α*-Cyperone mitigated OGD-induced cardiomyocyte inflammation and oxidative stress. Cardiomyocytes were treated with different concentrations (15, 30, and 60 *μ*M) of *α*-cyperone for 24 hours after OGD induction. (a) The profiles of inflammatory cytokines were assessed by qRT-PCR. (b) The expression of inflammatory response proteins was examined by WB. (c) The MDA content and (d) SOD activity were evaluated by colorimetry. (e) ROS production was determined with the ROS detection kit. All experiments were repeated three times and data were expressed as mean ± SD; ^∗∗∗^*P* < 0.001 (vs. CON), ^∗∗∗∗^*P* < 0.0001. ^&^*P* < 0.05 (vs. OGD), ^&&^*P* < 0.01, and ^&&&^*P* < 0.001.

**Figure 3:** *α*-Cyperone inactivated the Akt/FOXO3a/NF-*κ*B pathway in OGD-treated cardiomyocytes. Cardiomyocytes were treated with *α*-cyperone (60 *μ*M) for 24 hours after OGD induction. (a) Expression of p-Akt, Akt, p-FOXOa3, FOXOa3, p-NF-*κ*B, and NF-*κ*B was monitored by WB. (b) Nuclear translocation of Akt, FOXOa3, and NF-*κ*B was assayed by cellular immunofluorescence. All experiments were repeated three times, and the data were expressed as mean ± SD. ^∗^*P* < 0.01 (vs. CON). ^&^*P* < 0.05 (vs. OGD), ^&&^*P* < 0.01.

**Figure 4:** Inhibition of Akt curbed the protective effect of *α*-cyperone against OGD-induced myocardial injury. After treatment of OGD-induced cardiomyocytes with *α*-cyperone (60 *μ*M) for 24 hours, the Akt inhibitor MK-2206 was added. (a) The viability of cardiomyocytes was assessed with the CCK-8 assay. (b) Cardiomyocyte apoptosis was examined by flow cytometry. (c) The profiles of apoptosis-related proteins were assessed by qRT-PCR. (d) The expression of inflammatory factors was tested by qRT-PCR. (e) Expression of inflammatory response proteins was checked by WB. (f) Detection of the MDA content and SOD activity was implemented by the colorimetric assay. (g) The ROS production was evaluated by the ROS assay kit. All experiments were repeated three times, and the data were expressed as mean ± SD. ^∗^*P* < 0.05 (vs. OGD), ^∗∗^*P* < 0.01, and ^∗∗∗^*P* < 0.001. ^&^*P* < 0.05 (vs. OGD+*α*-cyperone (60 *μ*M)), ^&&^*P* < 0.01.

**Figure 5:** Attenuating Akt activated the FOXO3a/NF-*κ*B pathway. After treatment of OGD-induced cardiomyocytes with *α*-cyperone (60 *μ*M) for 24 hours, the Akt inhibitor MK-2206 was added. (a) Expression of p-Akt, Akt, p-FOXOa3, FOXOa3, p-NF-*κ*B, and NF-*κ*B was gauged by WB. (b) Phosphorylation of Akt, FOXOa3, and NF-*κ*B was determined by cellular immunofluorescence. All experiments were repeated three times, and the data were expressed as mean ± SD. ^∗^*P* < 0.05 (vs. OGD), ^∗∗^*P* < 0.01, and ^∗∗∗^*P* < 0.001. ^&^*P* < 0.05 (vs. OGD+*α*-cyperone (60 *μ*M)).

RETRACTED

**Figure 6:** NF-*κ*B inhibition counteracted the protective effect of *α*-cyperone on OGD-mediated myocardial injury. After treatment of OGD-induced cardiomyocytes with *α*-cyperone (60 *μ*M) for 24 hours, the NF-*κ*B inhibitor Bay 11-7082 was added. (a) Cardiomyocyte viability was assayed with CCK-8. (b) Cardiomyocyte apoptosis was examined by flow cytometry. (c) Expression of apoptosis-associated proteins was gauged by WB. (d) qRT-PCR assessed the relative expression of inflammatory factors. (e) Expression of inflammatory response proteins was monitored by WB. (f) MDA levels and SOD activity were checked by the colorimetric assay. (g) ROS production was gauged using a ROS assay kit. All experiments were repeated three times and data are expressed as mean ± SD; ^∗^*P* < 0.05 (vs. OGD), ^∗∗^*P* < 0.01, and ^∗∗∗^*P* < 0.001.

## Data Availability

The data sets used and analyzed during the current study are available from the corresponding author on reasonable request.
